RETRACTED

# Facility Layout Optimization of Urban Public Sports Services under the Background of Deep Learning

**DOI:** 10.1155/2022/1748319

**Published:** 2022-07-18

**Authors:** Tieying Huang

**Affiliations:** Department of Physical Education, Xi'an University of Finance and Economics, Xi'an, Shaanxi 710100, China

## Abstract

The spatial layout and optimization of social facilities for sports are related to many factors such as urban economy, transportation, population, and urban planning. With the rapid development of artificial intelligence today, deep learning came into being. It also provides a lot of methods for our in-depth research on it. To solve the problem of unbalanced layout of urban social facilities for sports and the difficulty in meeting the needs of residents under the current background, this paper adopts the methods of M-P model, loss function, and activation function. Taking Hangzhou, a sports city that is about to host the Asian Games, as an example, it carried out an experiment to optimize the layout of urban public sports services. Through various tests and data, it divides the accessibility level of social facilities for sports in Hangzhou into four levels: high accessibility point (1.0-1.5), high accessibility point (0.5-1.0), the accessibility is average (0.2-0.5), and the accessibility is poor (<0.2). It also concluded that the areas with high accessibility (1.0-1.5) are Shangcheng District and Binjiang District, and the layout of sports facilities is optimal. According to the minimum facility point model, Xiaoshan District and Yuhang District need to add 6 large-scale social facilities for sports. Through this experiment, this paper can also provide a reference for other urban layouts. This has significance for the optimization of sports facilities and the optimization of public facilities.

## 1. Introduction

Deep learning takes the raw form of the data as input to the algorithm. It is represented by the algorithm that abstracts the original data layer by layer into the final feature representation that required by its own task and finally ends with the mapping of features to task goals. From the original data to the final mission goal “all-in-one go,” there is no human operation involved. In addition to model learning, deep learning also involves task modules such as feature learning and feature abstraction. It completes the final learning task with the help of multilayer task modules.

The population size of the city determines that its demand for social facilities for sports presents the characteristics of multilevel, multisystem, and multipattern. It is both viewing and engaging. It has become an important activity in modern society and needs the support of urban space. Especially, large cities need to be people-oriented, study the needs of the public for physical exercise, and plan the layout of social facilities for sports to improve urban functions and meet the increasing leisure and fitness needs of the people.

RETRACTED

However, due to the limitations of the sports system and the influence of unbalanced economic development, the construction of sports facilities in many cities has generally lagged behind for a long time. Coupled with poor management, urban large-scale sports facilities often have problems such as low utilization rates and low economic benefits. To solve the problem of unbalanced distribution of social facilities for sports and insufficient scale of sports facilities, especially in grass-roots communities, this paper studies the layout optimization of urban public sports service facilities based on deep learning. The innovation of this paper is that it can not only enrich and improve the existing theoretical system through this research, but also play a reference and comparison role for special planning of public service facilities. At the same time, it can also provide space guarantee measures for the development and exploration of sports industrialization.

## 2. Related Work

Neural network is a hierarchical system composed of many nonlinear computing units (or neurons, nodes). Chen proposed a novel deep learning framework to incorporate features so that the highest classification accuracy can be achieved with the information he needed. As a deep learning architecture, his stacked autoencoder can obtain useful high-level features [1]. However, the architecture he proposed was too simple and required more in-depth research to deal with complex situations. Shen introduced deep learning models for image registration, anatomical and cellular structure detection, tissue segmentation, computer-aided disease diagnosis, and prognosis. This helps to identify, classify, and quantify patterns in medicine and other fields [2]. Matthew proposed a deep learning application of hierarchies of hidden variables to build nonlinear high-dimensional predictors. He developed and trained deep learning architectures for spatiotemporal modeling. He trained deep architectures through stochastic gradient descent and parameter-regularized dropout, and achieved minimal error in minimizing out-of-sample predictions [3]. He utilized deep learning approximate message passing (LDAMP) networks. This neural network can learn the channel structure and estimate channels from a large amount of training data. Furthermore, he provided an analytical framework on the asymptotic performance of channel estimators [4]. His research provided a reference for other researchers, but the scope of application was too narrow and needs further improvement. In terms of urban public sports services, many researchers have already dabbled in it. Zi pointed out that with the increasing demand for community sports and public services, physical exercise in urban public areas has become the main means for most residents. His research has provided a lot of convenience for us to build a community sports public service system [5]. As public health construction is developing rapidly, the provision of public sports services at this phase is gradually diverging from the needs of residents. Ma used the fuzzy analytic hierarchy process to construct and verify the optimization model of public sports services. The indicators of his optimization model have good applicability [6]. However, in terms of actually meeting the needs of residents, the practicality of his model is still lacking. It still needs to be further adjusted to actually match the needs of residents. Chen proposed an optimization-inspired deep learning inversion solver to quickly solve various problems encountered in analyzing public service data [7]. However, in terms of the actual layout of social facilities for sports, his method lacks certain guidance, and it needs to cooperate with the algorithms studied by other predecessors to achieve better results.

RETRACTED

## 3. Deep Learning Algorithm for the Layout of Urban Social Facilities for Sports

Deep learning has developed to this day. To sum up, its origin can be attributed to two different approaches: perceptron and Boltzmann machine. Deep learning, which originated from perceptrons, combines multiple perceptrons together to obtain a multilayered perceptron. On the basis of multilayer perceptron, coupled with the convolutional neural network similar to the structure of the human visual cortex, it is widely used in image recognition [8]. This is a supervised learning. It trains the network by continuously correcting the difference between the actual output and the desired output. Deep learning, which originated from restricted Boltzmann machines, is a type of unsupervised learning. It only trains the network on specific training data. Boltzmann machines are based on graphical models. Combining multiple restricted Boltzmann machines can get deep Boltzmann machines and deep belief networks.  Figure 1 shows the principles involved.

### 3.1. M-P Model

The M-P model is an artificial network model that mimics biology. It can perform calculations on complex data using three parts including network structure, connection weights, and learning ability. In the M-P model, there are multiple inputs {*x*|*i* = 1, 2, ...., *n*}, and after the operation, an output *y* is generated. The operation part includes weighted accumulation and threshold judgment. The M-P model stipulates that the input and output signals are all binary signals, that is, 0 or 1 [9]. Each input *x*_*i*_ is multiplied by the corresponding connection weight w_*i*_ and added to get the activation value:

(1) $$\begin{array}{c} M-P=\sum_{i=1}^{n}w_{i}x_{i}. \end{array}$$

Each input signal has a connection weight that represents how important that input signal is compared to other input signals [10].

(2) $$\begin{array}{c} \sum_{i=1}^{n}w_{i}x_{i}-h\geq 0. \end{array}$$

However, since it may be an arbitrary value, not 0 or 1 as defined by the M-P model, a function called an activation function is also required to transform this arbitrary value so that its output value is 0 or 1 [11]. It can be seen that the activation function is both a discriminator of the threshold and a normalizer of the output value:

(3) $$\begin{array}{c} \sum_{i=1}^{n}w_{i}x_{i}\left[0,1\right]=h. \end{array}$$

The activation function used by the M-P model is a step function. If the activation value is greater than the threshold *h*, it outputs 1; otherwise it outputs 0. The mathematical expression summed up is

(4) $$\begin{array}{c} y=f\left(\sum_{i=1}^{n}w_{i}x_{i}-h\right),\\ y=f\left(\sum_{i=1}^{n}w_{i}x_{i}-h\right)=\left\{1\text{if}\sum_{i=1}^{n}\begin{array}{c} w_{i}x_{i}-h\geq 0\\ w_{i}x_{i}-h\leq 0. \end{array}\right.. \end{array}$$

The M-P model uses a step function, also known as a threshold activation function. As can be seen from this model, the threshold discriminator is a boundary decision hyperplane. If the value is above this boundary decision hyperplane, the output value is 1. If it is below the boundary decision hyperplane, the output value is 0 [12]. The M-P model can realize three logical operations of NOT and AND.

(5) $$\begin{array}{c} \sum_{i=1}^{n}w_{i}x_{i}-h=0. \end{array}$$

As shown in the above formula, taking *w* = 1, *h* = 0.5, the model realizes the NOT operation.

(6) $$\begin{array}{c} f\left(-x+0.5\right)=\left\{\begin{array}{cc} 1, & \text{if}x=0,\\ 0, & \text{if}x=1. \end{array}\right. \end{array}$$

In this formula, taking *M*1 = *W*2 = 1, *h* = 0.5, the model realizes the OPERATION. It then takes *m* = *w*_2_ = 1, *h* = 1.5, and the model implements AND operation.

(7) $$\begin{array}{c} f\left(x_{1}+x_{2}-1.5\right)=\left\{\begin{array}{cc} 1, & \text{if }x_{1}=1\text{ and }x_{2}=1. \end{array}\right.. \end{array}$$

However, the M-P model cannot implement the XOR operation. If the two values are different, the result is 1. If the two values are the same, the result is 0. The role of the perceptron is to complete the classification and recognition of external inputs [13]. If the external input is linearly separable, a single-layer perceptron must be able to separate it into two categories. Structurally, the single-layer perceptron is the same as the M-P model. However, the difference between the two is essential. The connection weight parameter *w* and the threshold *h* of the model are preset and cannot be changed. The connection weight parameter *w* and the threshold *h* of the perceptron can be automatically corrected by training [14]. Although the perceptron has the ability to learn, it cannot solve the simple linear inseparable distribution problem in the two-dimensional plane. The judgment basis of the perceptron output value is still the boundary decision plane. This is a linear plane and cannot handle linearly inseparable cases. As shown in Figure 2, the classification can be carried out only when the decision plane is used as a classification tool from linearly separable to inseparable cases.

RETRACTED

In this paper, the author designed Faster *R* to speed up and simplify the conventional model to set up the experiment. Its conception is very delicate, and the process is more compact. Moreover using the largest network, the accuracy of PASCAL VOC 2007 is small, ranging from 66% to 67%.

Compared with other algorithms, it does not change the target candidate region generation and uses the selective search algorithm. The difference is that the author sets a region of interest algorithm for it. It maps candidate regions onto feature layers. It directly extracts deep features from regions on the feature layer, which avoids constantly inputting parts of images from different regions. It directly uses the extracted features to predict the region category with softmax and uses the network to learn a bounding box regressor. It organizes the entire feature extraction, classification, and boundary regression into one part, which improves the efficiency of the entire model.

Faster *R* overcomes the disadvantage of redundant operations when extracting features. It unifies feature extraction, classification, and bounding box regression for object detection into one box. It has good results in both speed and accuracy. However, the inefficient extraction of candidate regions with Faster *R* is still a bottleneck. Because the first step in detecting object locations is to generate a stack of potential bounding boxes or regions of interest. These are generated through selective search, which is time-consuming and difficult to incorporate into GPU operations.

In Faster *R*, a region generation network is introduced, which makes the candidate region extraction very efficient. It combines the extraction of candidate regions with the target detection network in Faster *R*, so that target detection can be achieved in the same network, which greatly improves the detection speed. The basic structure of Faster *R* network is shown in Figure 3.

RETRACTED

### 3.2. Loss Function

For the same structure, if the network parameters (weights and thresholds) are different, even if the input is the same dataset, the achieved output results are clearly different [15]. These different output values have advantages and disadvantages. Naturally, what we are looking for is the set of parameters that make the output value the closest to the expected value [16]. In principle, any function that can calculate the difference between the actual output value and the expected output value can be used as a loss function [17].

(1) For multiclassification problems (n training data are divided into *m* classes), the cross-entropy loss function is generally used:
  (8) $$\begin{array}{c} E=-\frac{1}{n}\sum_{i=1}^{n}\sum_{j=1}^{m}\gamma_{ij}1n\gamma_{ij}. \end{array}$$
(2) For recursive problems, a mean square (least squares) loss function is usually used:

(9) $$\begin{array}{c} E=\frac{1}{2}\sum_{i-1}^{n}{\left(\gamma_{i}-\gamma_{i}\right)}^{2}. \end{array}$$

The mean square loss function is widespread and easy to understand, and BP networks usually use it. The coefficient 1/2 is for the convenience of calculation. The sum of squares of the least squares method is to avoid the algebraic sum of the error values from the positive and negative cancellation that affects the actual sum of the error values. The actual output value of the network is a value between 0 and 1 calculated by the activation function.

For any random variable *X*, its information entropy is

(10) $$\begin{array}{c} H\left(X\right)=-\sum_{x\in \chi }P\left(x\right)\log P\left(x\right). \end{array}$$

It is to multiply the probability value of each possible item by the amount of information contained in the possible item and then accumulate to ensure a positive value. The cross-entropy error function is defined as

(11) $$\begin{array}{c} E=-\sum_{k}\gamma_{k}1n\gamma_{k}. \end{array}$$

The smaller the cross-entropy error value, the better the result. The larger the cross-entropy error value, the worse the result. Looking at the situation where the training data are divided into N groups, the cross-entropy error is

(12) $$\begin{array}{c} E=-\frac{1}{N}\sum_{k}\gamma_{nk}1n\gamma_{nk}. \end{array}$$

Loss functions are tools for tuning network parameters. The parameter values are usually fine-tuned, so one should think of the derivative of the loss function with respect to the parameter value W (weight). The positive, negative, and 0 values of the derivative value of the loss function with the parameter can indicate the direction of parameter change to ensure the gradual convergence of the loss function.

(13) $$\begin{array}{c} \left\{\begin{array}{cc} \text{if }\frac{\partial E}{\partial w}\leq 0, & \text{then }w↑,E↓,\\ \text{if}\;\frac{\partial E}{\partial w}\geq 0, & \text{then }w↓,E↓. \end{array}\right. \end{array}$$

RETRACTED

### 3.3. Activation Function

Activation function is responsible for the nonlinear transformation of the input signal, can fit various curves, and output the final result [18]. If it is not processed by the activation function, the input of each layer of the neural network is a linear function of the output of the upper layer. It is easy to verify that no matter how many layers the neural network has, the output is a linear combination of the inputs. Networks are only able to express linear maps. At this point, even if there are more hidden layers, the entire network is equivalent to a single-layer neural network. Therefore, the activation function provides the nonlinear modeling capability of the network.

The term activation in the activation function refers to whether a neuron in the network is activated by the sum of all input signals received. In other words, whether the signal received by this neuron works or is ignored. The activation function takes all inputs of the neuron, including input values and connection weights, through algebraic operations to obtain a comprehensive activation value. The activation function determines the value of the neuron with output 0∼1 or −1∼1 according to the distance between the activation value and the threshold [19]. Not any function is suitable for the activation function of neurons.

#### 3.3.1. Step Function

The M-P model and the perceptron use the following step function as the activation function.

(14) $$\begin{array}{c} f\left(x\right)=\left\{0\;\text{if}\sum_{i=1}^{n}\begin{array}{c} w_{i}x_{i}-h\leq 0\\ w_{i}x_{i}-h\geq 0. \end{array}\right.. \end{array}$$

#### 3.3.2. ReLU Function

The activation function ReLU is a very simple function, but it has no simple effects. The modified linear unit ReLU can be defined as

(15) $$\begin{array}{c} f\left(x\right)=\left\{\begin{array}{cc} 0, & \text{if}\;x\leq 0,\\ x, & \text{if}\;x\geq 0. \end{array}\right. \end{array}$$

That is, if the input value is greater than 0, it will output the value directly; otherwise it will output 0. Clearly, the role of the ReLU function is that when *x* > 0, *f*(*x*) > 0, the model will update the parameters; otherwise it will not be updated. This derivative function is a standard step function [20].

(16) $$\begin{array}{c} f\left(u\right)=\frac{1}{1+e^{-u}},\\ u=\sum_{i=1}^{n}w_{i}x_{i}-h. \end{array}$$

It is not difficult to see that the ReLU function calculation is clearly simple, and there is no gradient problem. Compared with sigmoid and tanh, ReLU converges 6 times faster. The ReLU function solves the problem of vanishing gradient and computational efficiency.

RETRACTED

#### 3.3.3. Derivative Function of ReLU Function

Since the gradient of the function ReLU is 0 when *x* < 0, this neuron may never be activated by any data again. As shown in Figure 4, the three functions all improve the negative end of the function ReLU, so they all belong to the derivative functions of ReLU [21].


(17) $$\begin{array}{c} y=f\left(v\right)\\ =\left\{\begin{array}{cc} x, & \text{if}\;x\geq 0,\\ ax, & \text{if}\;x\leq 0. \end{array}\right. \end{array}$$

Its derivative is

(18) $$\begin{array}{c} f^{\prime }\left(x\right)=\left\{\begin{array}{cc} 1, & \text{if}\;x\geq 0,\\ a, & \text{if}\;x\leq 0. \end{array}\right. \end{array}$$

When *x* < 0, the leaky ReLU function multiplies the variable by a small constant a, such as *a* = 0.01, so that a positive gradient of 0.01 can be obtained, thereby avoiding the problem of dead neurons. In PReLUfunction *y*=max(*ax*, *x*), a is a hyperparameter, not a fixed value. It is calculated by the error back-propagation algorithm. It is theoretically more reasonable than the leaky ReLU function.

## 4. Experiments on the Optimization of the Facility Layout of Urban Public Sports Services

Urban social facilities for sports shall be arranged according to scale and grade. It should not only meet the needs of large-scale events and large-scale sports events, but also focus on serving the national fitness movement. This enables citizens to exercise nearby, improves the utilization efficiency of grass-roots facilities, and achieves the effects of better accessibility, better social benefits, and better economic benefits [22]. Generally speaking, the classification of the layout of social facilities for sports in big cities should adopt the three-level standard configuration of municipal, district, and community levels. Municipal and district-level social facilities for sports mainly focus on competitive sports, host events, and daily serve the national fitness. The community level is a sports facility around the residents, which needs to meet the needs of community residents for exercise and fitness.  Figure 5 shows the service layout and requirements for a standard municipal sports facility.

Next, the author conducts the experiments in this section with the Chinese city of Hangzhou, which will host the 2022 Asian Games as the research object. As a city hosting large-scale sports events, in terms of public sports services, it must not only provide a large number of professional sports facilities services in a short period of time, but also provide an excellent sports facility layout for the vast population in daily life. Hangzhou is a new first-tier city in China, with an average annual GDP exceeding one trillion yuan and a permanent population of over 12 million. This can provide a good example for other cities in the layout of social facilities for sports.

RETRACTED

### 4.1. Accessibility Analysis of Social Facilities for Sports Based on GIS

With the continuous development of accessibility theory, it has been widely used in many research fields such as urban planning, transportation, education, medical care, shopping malls, and the layout and location of emergency and disaster relief points.

It analyzes the basic configuration of China's social facilities for sports. Regarding the spatial layout of Hangzhou's social facilities for sports and the service functions of social facilities for sports, there is still no more accurate and objective judgment on whether the principles of fairness and efficiency are reflected.  Table 1 shows the basic indicators of social facilities for sports in big cities.

To match this indicator, Hangzhou City implements the “National Fitness Program Outline” issued by the Chinese government. It has built a part of social facilities for sports through the annual investment of the sports lottery public welfare fund. This level of social facilities for sports has a strong “debt repayment” nature for the unbalanced development of competitive sports and mass sports in China for a long time [23]. By the end of 2020, Hangzhou will have fitness paths (3,849 fitness paths), fitness gardens (173), and fitness sports (more than 7,000). Its configuration is standard for fitness garden points: the fitness path is equipped with 20 sets of equipment, the fitness garden is equipped with 12 sets of equipment, and the fitness point depends on the space configuration.  Table 2 shows the service configuration of social facilities for sports in 8 different areas of Hangzhou.

Therefore, the layout characteristics of Hangzhou's public sports facilities are as follows: it “sees the needle” around the community and streets, it lacks unified planning, and sports facilities and equipment are mainly simple, safe, and durable. Although the exercise conditions of urban residents have been improved, it can meet the needs of some urban residents (the elderly) for physical exercise, but it cannot represent the level of sports development in a city. Therefore, this study uses GIS technology to further study the accessibility issues in the spatial layout of large-scale social facilities for sports in Hangzhou.

RETRACTED

#### 4.1.1. Determination of Starting Point and Destination

This study uses 71 large-scale social facilities for sports distributed in eight administrative districts of Hangzhou as the destination (point of interest) for residents' activities. It starts from 5,608 residential areas in Hangzhou to measure the accessibility of various residential areas in Hangzhou to large-scale sports facilities. Using crawler software, the starting point and destination of this study were obtained, and then all data were imported into ArcGIS system.

#### 4.1.2. Service Areas of Social Facilities for Sports

The service area of social facilities for sports refers to the set of areas that can be reached (i.e., reachable coverage area) after a certain time or a certain distance along the urban road network starting from a specific sports venue [24]. Therefore, it requires the area and scope of service that can be provided after a certain time distance. Well, it first needs to determine the speed at which citizens travel. This travel speed is determined by the mode of transportation chosen by city residents, such as walking, cycling, public transportation, and driving. The travel speed of Hangzhou citizens determined in this study is 40 km/h on average with the driving speed and with riding at an average speed of 15 km/h. The average walking speed is 10 km/h. Then, the average speed of the three travel modes of citizens is 21 km/h. According to the requirements of residents' 15-minute fitness circle, this study uses time Minutes (minutes) as the impedance unit. It uses three time impedances of 15 minutes, 30 minutes, and 60 minutes to calculate the scope of the service area of social facilities for sports in Hangzhou. Finally, it generates the service area of large social facilities for sports in Hangzhou by using the service area analysis layer in the ArcMap network analysis module. The calculation results are shown in Figure 6.

It can be clearly seen from Figure 6 that, in the impedance units of 15 minutes, 30 minutes, and 60 minutes, the spatial distribution of large-scale social facilities for sports in Hangzhou is regionally uneven. In the 15-minute impedance unit, large-scale social facilities for sports are mainly concentrated in the lower and upper old towns. The maximum total is more than 12, which has a lot to do with the geographical location of their centers. The 30-minute and 60-minute impedance unit results have the same trend. The density of the spatial distribution of social facilities for sports follows the decreasing law of the old city-new city-new development zone. Among them, the highest is the West Lake District, with a total of 5. The lowest belongs to Yuhang District, with a total of 1. Divided by region, at present, large-scale social facilities for sports are mainly distributed in the main city. Jiangnan City and Xiasha City, which are two subcity areas, have almost no distribution in the “six major groups.”

RETRACTED

The sports service area only considers the relationship between social facilities for sports and the road traffic system. It does not take into account the demographic factors of urban residents' physical exercise needs and the living and living location factors of those with physical needs. Therefore, on the basis of the analysis of the service area of social facilities for sports, this study carried out the accessibility calculation of large-scale social facilities for sports in Hangzhou.

### 4.2. Accessibility Calculation of Social Facilities for Sports

The accessibility calculation in this study is done in two steps. First, it needs to calculate the shortest time (distance) from all origins to the destination. It refers to the shortest time (distance) for all people with physical exercise to reach all large sports and social facilities starting from where they live. On this basis, it uses a potential model to calculate the accessibility of each community point to large sports facilities in Hangzhou.

#### 4.2.1. Calculation of the Shortest Distance

There is an important model in the model of network analysis module, namely, OD matrix model. Due to the fast operation speed of the OD matrix model, the shortest paths between multiple origins and multiple destinations on the road network can be obtained through it. Therefore, people often use it to solve multiorigin and multidestination shortest path problems. First, it creates a new OD cost matrix in the location allocation module of ArcGIS 10.2 and then opens the network analysis window. The starting point is loaded as 5608 districts in Hangzhou, and the destination is loaded as the selected 71 large-scale social facilities for sports in Hangzhou. It usually has time or distance as an impedance condition in its analysis settings in the OD matrix. In this study, the transit time is used as the impedance, and each result is listed correspondingly in the attribute table of this layer. The results are shown in Figure 7.

It can be seen from the OD matrix in Figure 7 that the sports facilities and the community are not much different from the top, bottom, left, and right of the OD curve, and most of the time they are below the OD curve. The calculated value of 71 sports facilities is generally lower than that of the community, with the lowest value being only 10. However, the highest point basically coincides with the distribution of the cells, and the peak value is 86, which is juxtaposed under the OD curve. The shortest travel time from large social facilities for sports to residential communities is an important basis for judging the accessibility of facilities. The calculation of the shortest transit time ignores the service capacity of public sports facilities (the size of the facility, the number of sports events that can be carried out, etc.). Therefore, on the basis of calculating the shortest transit time, the potential model can be used to describe the accessibility of large-scale social facilities for sports in Hangzhou more comprehensively.

RETRACTED

#### 4.2.2. Potential Model Analysis Process

The potential model was first proposed in the research on the accessibility of medical service facilities. Since then, it has been widely used in the research of public service facilities (medical, school, fire emergency, etc.). The potential model formula is as follows:

(19) $$\begin{array}{c} A_{i}=\sum_{j=1}^{n}A_{ij}\\ =\sum_{j=1}^{n}\frac{M_{j}}{D_{ij}}. \end{array}$$

*A*_*i*_ is the sum of the potentials of *n* discretely distributed objects for point *i*, *M*_*j*_ is the scale of point *j*, and *D*_*ij*_ is the impedance (time or distance) between point *j* and point *i*. Through the research and development of scholars, it has broken through the constraints of the distance index dimension in formula (19), introduced the friction coefficient *β*, and formed the potential model of geography, which is also the model adopted in this study. The potential model formula is as follows:

(20) $$\begin{array}{c} A_{i}=\sum_{j=1}^{n}\frac{M_{j}}{D_{ij}^{\beta }}. \end{array}$$

*A*_*i*_ is the accessibility measure of community point *i*; *M*_*j*_ is the service capacity of large public sports facility *j*; *D*_*ij*_ is the shortest time or distance from community point *i* to large public sports facility *j*; *β* is the impedance coefficient. After literature review, this study will determine the service capacity of sports facilities through population density and the number and type of points of interest. The formula looks like this:

(21) $$\begin{array}{c} M_{j}={\text{Log}}_{10}\left\{F_{j}{\left(\sum_{i=1}^{n}w_{i}p_{i}\right)}^{q}\right\}. \end{array}$$

Among them, F_j_ is the population density, *n* is the type of POI, *W*_*i*_ is the influence factor of POI *i*, P_i_ is the number of POIs for the type of POI, and *q* is the correlation coefficient. All large social facilities for sports were set as points of interest of the same type in this study. Therefore in formula (21), both *n* and *W*_*i*_ are 1. It obtains the formula for calculating the service capacity of large-scale social facilities for sports:

(22) $$\begin{array}{c} M_{j}={\text{Log}}_{10}\left(F_{j}P^{q}\right). \end{array}$$

Then, the shortest time from the residential area to the large-scale sports facilities obtained by the service capacity is brought into the potential model formula, to calculate the accessibility of each residential area to the large-scale sports facilities.

RETRACTED

#### 4.2.3. Result Expression and Analysis of Accessibility

The accessibility results of social facilities for sports in Hangzhou City are calculated by the formula, and then it needs to use spatial interpolation analysis (IA) technology to express the obtained accessibility results in space. This can more intuitively show the accessibility of each area. The interpolation methods often used in GIS software are inverse distance weighting method, spline function method, and kriging method. In this study, the kriging method is used for spatial interpolation because it can both have the function of predicting the surface and provide some measure of the certainty or accuracy of the prediction.

As shown in Figure 8, according to the accessibility measures of large-scale social facilities for sports in Hangzhou, the accessibility level of social facilities for sports in Hangzhou can be divided into four levels: high accessibility points (1.0-1.5), high accessibility point (0.5-1.0), average accessibility point (0.2-0.5), and poor accessibility point (<0.2). It can be seen from Figure 8 that the areas with high accessibility (1.0-1.5) are Shangcheng District and Binjiang District, with 4.8 and 5.1 points, respectively. This is related to the intensity of the construction of sports facilities in these two regions under the policy. Other regions performed fairly well in the middle range. However, among the points with poor accessibility (<0.2), Jianggan District and Yuhang District accounted for the most points, 5.1 and 5.2, respectively. This is related not only to policy compliance, but also to the more partial geographical location of the two regions.

### 4.3. Optimization of the Layout of Social Facilities for Sports in Hangzhou

Since urban social facilities for sports are inseparable from the daily life of urban residents, it is the goal of the layout of social facilities for sports to rationally distribute social facilities for sports and meet the needs of residents for physical exercise as much as possible. In the specific layout and optimization of social facilities for sports, it is necessary to consider not only the use efficiency of sports facilities, but also the fairness that all urban residents can enjoy the social facilities for sports equally. However, the different emphases on the use efficiency and fairness of the layout of social facilities for sports will lead to different layout characteristics (large-scale centralized and small-scale decentralized) of urban social facilities for sports. Therefore, the layout and optimization of social facilities for sports should take both fairness and efficiency as the main principle.

RETRACTED

According to the shortest time in Figure 9, it can be concluded that the average time from each living quarter to its nearest sports facility is 15 minutes. This aligns with the proposed 15-minute fitness circle goal. Therefore, in this study, the impedance time of the minimum impedance analysis of sports facilities in Hangzhou is 15 minutes, the existing 71 large-scale sports public facilities are selected as the destination, and the 5608 communities in Hangzhou are the request points. Although the average time from a community to the nearest sports facility is 15 minutes, there are still a large number of living quarters in the city that cannot reach large sports public facilities within 15 minutes. Among them, the central urban areas (Shangcheng District, Xiacheng District, Gongshu District, Jianggan District) are in good condition due to the dense sports facilities. Most communities can reach sports facilities in 15 minutes or less. In the southwest and northeast of Yuhang, and the southern part of Xiaoshan, there are a large number of residential areas, which cannot be reached within the specified time due to the lack of large-scale social facilities for sports. There are also the northwest and central parts of Yuhang and the southeast of Xiaoshan. Due to road reasons, it is impossible to reach the sports facilities within the specified time. The two districts of Yuhang and Xiaoshan need to strengthen the construction of sports public facilities and the repair of roads, so that the service scope can cover the entire administrative area with the maximum extent.

In addition, according to the minimum facility point model, Xiaoshan District and Yuhang District need to add 6 large-scale social facilities for sports. The results are shown in Table 3. The selection of optimization methods should be viewed from the general optimization methods of urban public service facilities. It is usually divided into three types: establishing a new distribution system of public service facilities; building new service facilities on the basis of existing public service facilities; and renovation and reconstruction of some existing service facilities with poor service capabilities. However, the distribution system of urban social facilities for sports is the product of historical accumulation and the inertia of urban development. In particular, large-scale social facilities for sports in cities are different from other types of public service facilities (such as hospitals and schools) and can be completed by overall relocation. Therefore, when optimizing the layout of sports facilities in this study, it is mainly based on the combination of adding new social facilities for sports and improving existing sports facilities to optimize the layout of urban social facilities for sports in Hangzhou.

RETRACTED

In addition, it is necessary to continue to improve the traffic and road conditions in various regions. After reorganizing the layout of Hangzhou's sports facilities, it can effectively meet the needs of residents outside the central area for large-scale social facilities for sports and improve the accessibility of Hangzhou's urban social facilities for sports as a whole.

Figure 10 shows the renovated sports facilities in Hangzhou for the Asian Games and the upcoming sports facilities for the Asian Games. According to Figure 10, we can conclude that Hangzhou takes Shangcheng District and Xiaoshan District as key new facility areas for the Asian Games, adding up to more than 11 areas. These two areas are also in line with the key areas that we have tested. The two areas with the most repaired sports facilities are Gongshu District and Xiaoshan District, adding up to 16, which is also in line with our calculation, indicating that our model is effective.

## 5. Conclusions

This paper adopts a variety of algorithms under the background of deep learning and fully considers the population differences of each residential area and the differences in the physical exercise needs of regional residents, and studies the layout of social facilities for sports. Due to the lack of academic ability and the difficulty of data collection (public transportation network data), this study failed to include all factors, resulting in a slightly less convincing analysis of existing problems. In the future, the authors will make up for these shortcomings through further research and at the same time look forward to using more methods to research the optimal solution for the layout of social facilities for sports, to provide convenience for the lives of residents.

## Figures and Tables

**Figure 1:** Perceptron and Boltzmann machine learning principles of deep learning.

**Figure 2:** Linearly separable and inseparable diagrams.

**Figure 3:** The basic structure of Faster R.

**Figure 4:** Schematic diagram of ReLU and its derivative functions leaky ReLU function.

RETRACTED

**Figure 5:** Service radius of social facilities for sports in big cities.

**Figure 6:** Distribution of service areas of large social facilities for sports.

**Figure 7:** OD cost matrix layer.

**Figure 8:** Spatial distribution of accessibility to large social facilities for sports.

**Figure 9:** Results of minimum impedance of sports facilities in Hangzhou.

**Figure 10:** Location of new sports facilities in Hangzhou.

**Table 1:** Basic indicators of social facilities for sports in big cities.

	Planning criteria	Audience scale	Land area	Per capita indicator
		Thousands	(ha)	(m)
Stadium	1/1 million-2 million	30–50	86–112	0.04-0.122
Gymnasium	1/1 million-2 million	4–10	11–20	0.0055-0.02
Swimming pool	1/1 million-3 million	2–4	13–17	0.0043-0.17
Shooting range	1/1 million-3 million	2–4	10	0.005-0.01
Total				0.0548-0.168

**Table 2:** The service capacity of large-scale social facilities for sports in 8 administrative districts.

Administrative area	Shangcheng area	Xiacheng area	Gongshu area	Jianggan area	Xihu area	Binjiang area	Xiaoshan area	Yuhang area
Population density (people/square kilometer)	18450	18625	12110	10468	9878	10129	8487	7874
Number of sports facilities	3	7	6	21	16	7	8	3
Service capabilities	4.74	5.12	4.86	5.34	5.2	4.85	4.83	4.37

**Table 3:** Additional sports facilities planning.

Program	Number	Service population	Land size (ha)
Municipal sports center	1	Total population of the city	30
Comprehensive gymnasium	1		8–12
Stadium	1		1–3
Shooting range	1		1–2
Other municipal single sports facilities	1		20

## Data Availability

The data underlying the results presented in the study are available within the article.
